This article has been retracted.

# Innovate a Standard for the Future Model of Nursing Care at Medical-Surgical Units in Najran University

**DOI:** 10.1155/2022/2959583

**Published:** 2022-07-20

**Authors:** Abeer Y. Mahdy Shalby, DaifAllah D. AlThubaity

**Affiliations:** ^1^Medical-Surgical Nursing Department, Faculty of Nursing, Najran University, Saudi Arabia; ^2^Pediatric Nursing Department, Faculty of Nursing, Najran University, Saudi Arabia

## Abstract

**Aim:**

Innovate a standard for the future model of nursing care at medical-surgical units in Najran University through a training program for the standard of the future model evaluation on studied nurses' knowledge, attitude about innovation standards, and innovative behavior among nurses.

**Methods:**

A quasi-experimental research was used to achieve the study's goal; the research was carried out at Najran University Hospital at Najran, in the medical and surgical units, as well as outpatient clinics. The sample is a convenience type; 100 nurses were used. *Tool*. A structured questionnaire sheet was used for data collection that includes nurses' knowledge, attitude, and individual innovative scale.

**Results:**

This reveals the studied nurses related to their individual innovative scale pre- and postintervention. Concerning resistance to change, the mean of them preintervention is *x* ® SD 9.08 ± 2.60. Concerning opinion leadership, the mean of them postintervention is *x* ® SD 14.32 ± 3.16. There is a highly significant difference (*p* < 0.01^∗∗^) preintervention as regards all domains listed.

**Conclusion:**

The educational program significantly enhances nurses' knowledge and attitude, according to our present study. Nurses' innovative skills are also improved by enhancing their knowledge and attitude. Before and after the educational program was implemented, there was a highly positive linear association between the nurses' knowledge, attitude, and innovative skills at *p* < 0.01.

## 1. Introduction

Nurses are critical to high-quality care, so healthcare would come to a stand without them. There is not a single intervention or healthcare program in which they do not play an important role [1, 2].

The innovation idea is nothing new to the profession of nursing. Nurses all over the world engage in new actions on a daily basis with the goal of improving healthy patient care results while minimizing costs. Numerous of these initiatives have resulted in considerable improvements in patients, nations, and all systems of healthcare. On the other hand, nursing support for healthcare innovation is rarely familiar, publicized, or shared through nurses and the broader public [3].

Innovation is often characterized as a new method device. “Practice” is described as a rule or custom of practicing; it is also described as follows: reduplicate action for getting expertise, the resulting state of being skillful, information put into action, and vocation performance. You can be innovative in a variety of ways, including being creative or solving issues to develop a new strategy, product, or service that others enjoy. Innovation is a novel way of doing something that is more effective or less expensive [4]. Doing things differently in order to achieve significant performance improvements is what innovation entails. Unlike popular belief, most discoveries do not come from laboratories, policymakers, or senior executives. Employees within those organizations develop the majority of inventions, whether in the public or private sector [5].

Nursing and nurses will not and cannot be free to innovate and improve practice in isolation as a result of transformation and change. There are successful and long-lasting innovations and changes in practice, despite the fact that nursing is a compound and difficult profession that requires well-informed, competent, and critical thinkers and doers, as well as a lot of enthusiasm, devotion, and hard work [6].

Nursing application innovation is critical for primary, secondary, and tertiary care, identifying and avoiding hazard factors, promoting good lifestyle attitudes, and assessing care and other techniques. This is because the institutions that employ them can generate and discover new information, methods, and services [7].

Nurses are devising innovative strategies to assist patients who are not receiving the care they require, such as making minute clinics more accessible, improving maternal and infant care, and altering treatment at the bedside. To deal with the problems of new technology as well as an out-of-control nursing shortage, a deeper understanding of how innovation works, what it looks like when people come up with new ideas, and how organizations can encourage or discourage it is required [8, 9].

## 2. Methods

### 2.1. Hypothesis

The hypotheses of the study are as follows:

*H^1^:* nurses' knowledge and attitude about innovation were improved postimplantation.

*H^2^:* nurses' knowledge and attitude about innovation standards had a positive effect postprogram implementation.

*H^3^:* nurses' knowledge and attitude had a positive effect on improving innovative behavior.

### 2.2. Research Design

To achieve the study's goal, a one-group pretest/posttest quasi-experimental research methodology was used. It is an empirical study that uses nonrandom assignment to estimate the effect of an intervention on its target population.

### 2.3. Setting

The study was carried out at Najran University Hospital at Najran, in the following departments: medical units, surgical units, and outpatient clinics.

### 2.4. Participant

Participants were recruited using a convenience sampling technique at Najran University Hospital at Najran, in the following departments: medical units, surgical units, and outpatient clinics. A total of 100 nurses, from the previously mentioned setting, who agreed to share in the study were recruited in the study. The study duration extended over a period of five months, from the 1^st^ of September 2021 to the end of January 2022.

### 2.5. Sample Size

The sample size was determined using a statistical power of 90%, a degree of confidence (1 − alpha error) of 95%, an alpha of 0.05, and a beta of 0.1. The sample size was set at 90 nurses. With a 15% sample attrition rate, the ultimate sample size is 100 nurses.

### 2.6. Tools of Data Collection

The current study's data were gathered using a structured electronic questionnaire sheet that the researcher created in English after researching literature reviews [10]. It is divided into four sections as follows:

*Part I:* concerned with the demographic profile of the studied nurses, it included sociodemographic characteristics of the studied nurses such as age, experience, qualification, nationality, and training courses.

*Part II:* concerned with nurses' knowledge, it included 14 MCQ questions such as the concept of innovation standard “2 items,” the benefits of innovation standard at nursing “3 items,” the factors affecting innovation standard at nursing “3 items,” the principal achievement of innovation standard strategy “3 items,” and the ways of achievement of innovation standards “3 items.” Each answer was scored with 1 if correct and zero if incorrect. The total knowledge score was divided into two categories such as unsatisfactory (<70.0%) and satisfactory (≥70.0%).

*Part III:* concerned with nurses' attitude, it included 6 questions such as “I think that innovation causes wasting time and effort and that innovation at nursing causes a huge load on nurses without benefits.” Each answer was scored on the Likert scale as follows: agree “3,” sometimes “2,” and disagree “1” for positive items and vice versa for negative points. The total attitude score was categorized as follows: negative attitude (<70.0%) and positive attitude (≥70.0%).

*Part IV:*concerned with the individual innovative scale, it will be adopted from [11]. To assess innovative behavior, it included 20 items divided into five domains such as opinion leadership, openness to experience, resistance to change, cautiousness, and risk-taking. Each answer was scored on the Likert scale as follows: agree “3,” sometimes “2,” and disagree “1” for positive items and vice versa for negative points. The total innovative score was categorized as follows: high (>70.0%), moderate (50 to 70%), and low (<50.0%).

### 2.7. Operational Design

#### 2.7.1. Preparatory Phase

A literature review, tool development, and testing of the validity and reliability of the study's generated tools were all part of this phase, including a review of previous and recent literature and studies relevant, as well as a familiarization with the many components of the study research problems using available books, periodicals, magazines, and articles. A statistician used Cronbach's alpha coefficient test in the SPSS program version 21 to split all questions on the instrument and compute all correlation values for them, ensuring that the constructed tool was reliable. It was carried out on 10% of the nurses tested (*n* = 10), with strong reliability for knowledge Cronbach′s = 0.849, attitude = 0.817, and innovative scale = 0.887.

#### 2.7.2. Pilot Study

A pilot research with a group of ten breastfeeding women was conducted. It is done prior to gathering data to assess the feasibility, time, cost, and adverse events of a full-scale research plan. The appropriate changes were made as a result. The sample included participants from the pilot research.

#### 2.7.3. Fieldwork

This phase started from August 2021 to March 2022; it included taking permission from the hospital director and explaining the aim to the director and head nurses; after that, take consent from them to collect data; after that, distribute the Google form in the hospital WhatsApp group to collect data; the session was divided into an orientation to the innovation standard. Feedback was given at each session, starting about the last one and finishing each session by summary; after that, the evaluation method was selected to suit the nurses' needs and achieve goals.

#### 2.7.4. Frame of the Study

The frame of the study was done through the following phases:

*Assessment phase:* assess nurses' knowledge, attitude, and innovative scale.

*Planning phase:* objectives, priorities, and expected outcomes will be established based on the findings to meet nurses' knowledge and innovative skills and needs.

*Implementation phase:* prepare appropriate media, such as brochures, for the new standard in nursing care throughout the implementation phase. The educational program was implemented in the previously specified environments. The instructional program consisted of four classes held once a week, each lasting 20 to 30 minutes. The first session concentrated on the notion and principles of innovation standards. The second session focused on the characteristics of the nursing innovation standard, as well as the methods and strategies for achieving the goal. The third session focused on the advantages and benefits of innovation in nursing. The fourth session focused on innovation directions for nurses.

*Evaluation phase:* reevaluate nurses' knowledge, attitude, and innovative skills after implementing the educational program, which were compared with pretest levels.

### 2.8. Ethical Considerations

The director of the previously described setting gave his assent to the research. After the researcher briefed each nurse about the study's goal, they signed a consent form. Furthermore, the nurse who volunteered to participate in the study was advised that all information acquired would be kept private. They also have the option to leave the study at any moment.

### 2.9. Statistical Analysis

Organize and categorize the data and display the results in tables. The Statistical Package for the Social Sciences was used to analyze the data on a compatible personal computer (SPSS Inc.; version 21; IBM Corp., Armonk, NY, USA). Means and standard deviations were used to present continuous variables. To compare the pre- and postintervention scores, the chi-square was used. A *t*-test is an inferential statistic that is used to see if there is a significant difference between two groups' means. The results were considered significant when the probability of error is less than 5% (*p* < 0.05) and highly significant when the probability of error is less than 0.1% (*p* < 0.001).

## 3. Results

As shown in Table 1, this study is conducted on 100 nurses. Regarding their characteristics, more than two-thirds of them (68%) range in age from 20 to less than 25 years old, with mean age *x* ® SD 25.26 ± 4.78 years. As regards their experience, more than half of them (54%) have less than one year, while 8% of them have more than five years. In addition, as regards their qualification, most of them (84%) have a bachelor's degree, while 6% of them have a diploma. The majority of them (92%) are Saudi Arabians. Also, nearly two-thirds of them (62%) have no training courses about innovation, but 38% of them have.

Table 2 illustrates the knowledge of the studied nurses about innovation standards pre- and postintervention. Most of them (86%) have a correct answer as regards the principle achievement of innovation standard strategy “3 items” postintervention, but 83% of them have an incorrect answer regarding the ways of achievement of innovation standards “4 items” preintervention. There is a highly statistically significant difference (*p* < 0.01^∗∗^) between pre- and postintervention as regards all features registered.

Figure 1 represents the studied nurses' total knowledge about innovation standards pre- and postintervention. Most of them (88%) have satisfactory knowledge postintervention, while more than three-quarters of them (76%) have unsatisfactory knowledge preintervention.

Table 3 reveals the studied nurses related to their individual innovative scale pre- and postintervention. Concerning resistance to change, the mean of them preintervention is *x* ® SD 9.08 ± 2.60. Concerning opinion leadership, the mean of them postintervention is *x* ® SD 14.32 ± 3.16. There is a highly statistically significant difference (*p* < 0.01^∗∗^) between pre- and postintervention as regards all domains listed.

Figure 2 shows the sample of nurses' individual innovative scale pre- and postintervention. More than half of them (52%) have high postintervention, while almost half of them (48%) have low preintervention.

Figure 3 clarifies that most of the studied nurses (84%) have a positive attitude about innovation postintervention, while more than two-thirds of them (68%) have a negative attitude preintervention.

Table 4 shows highly statistically significant positive correlations preintervention (*p* < 0.01^∗∗^) between the total knowledge and the individual innovative scale of the studied nurses (*r* = 0.601), between their total knowledge and their total attitude (*r* = 0.564), and also between their individual innovative scale and their total attitude (*r* = 0.537).

Table 5 shows highly statistically significant positive correlations postintervention (*p* < 0.01^∗∗^) between the total knowledge and the individual innovative scale of the studied nurses (*r* = 0.577), also between their total knowledge and their total attitude (*r* = 0.498), and between their individual innovative scale and their total attitude (*r* = 0.601).

## 4. Discussion

The current study revealed that there was a highly statistically significant differentiation (*p* < 0.01^∗∗^) before and after regarding all domains of knowledge- and attitude-related innovation standards. Moreover, most of them had satisfactory knowledge postintervention, while more than three-quarters of them had unsatisfactory knowledge preintervention. Furthermore, most of the studied nurses had a positive attitude about innovation postintervention, while more than two-thirds of them had a negative attitude preintervention. These results were attributed to the effective training program, which was prepared by the researcher dependent on nurses' needs detected by a pretest and which also used different illustrative teaching methods such as PowerPoint, videos, and attractive animations.

These results were supported by [12] which stated that the theoretical knowledge (88.4 vs. 81.7, *p* 0.001), operation skills (94.8 vs. 90.3, *p* 0.001), and total core competency score (156.2 vs. 148.8, *p* 0.05) were statistically substantially higher in the research group than in the control group. [13] stated that the nurses were enthusiastic about using modern technology, but there were obstacles such as a shortage of nurses, insufficient in-service training for staff on how to use the new technology, and a lack of electricity. [14] detected that there was an improvement in nurse managers' innovative managerial knowledge and skills, which then diminished at follow-up after three months of implementing the training program. Also, [15, 16] detected that nurses' knowledge, attitude, and performance in relation to ethical codes can all be improved through group reflection.

In addition, the current study demonstrated the studied nurses' individual innovative scale pre- and postintervention. More than half of them had high innovative skills postintervention, while almost half of them had low skills preintervention. Also, it was mentioned that it improved in the domains of the innovative scale.

These results were supported by [17, 18] which detected that after the training, nurses' self-rated innovation capacity (*p* 0.001, 95% confidence interval 12.79 to 15.05) and research ability (*p* 0.001, 95% confidence interval 14.39 to 19.09) both improved significantly. Also, [19, 20] revealed that empowering education can help nurses perform their jobs more effectively and master their professional abilities. [21] reported that to equip future generations of medical professionals with the ability to innovate efficiently and effectively, targeted education is required. Besides, [22] revealed that changing and improving nursing management staff's creativity affects their performance at Benha University Hospital. [23] stated that throughout the program, there was a statistically significant increase in the level of creativity and productivity among staff nurses.

Furthermore, the current study discovered highly statistically significant positive correlations between the total knowledge, the attitude, and the individual innovative scale of the studied nurses after intervention (*p* 0.01^∗∗^) at *p* value 0.01^∗∗^. These results agree with [24, 25] which showed that at the postintervention and follow-up program phases, there was a highly statistically significant positive link between the head nurses' managerial innovation knowledge, skills, and degree of professional competency.

## 5. Conclusion

The educational program significantly enhances nurses' knowledge and attitude, according to our present study. Nurses' innovative skills are also improved by enhancing their knowledge and attitude. Before and after the educational program was implemented, there was a highly statistically significant positive association between the nurses' knowledge, attitude, and innovative skills at *p* < 0.01.

## Figures and Tables

**Figure 1:** Distribution of nurses related to their knowledge about innovation standards pre- and postintervention (*n* = 100).

**Figure 2:** Distribution of nurses related to their individual innovative scale pre- and postintervention (*n* = 100).

**Figure 3:** Distribution of studied nurses related to their attitude level about innovation pre- and postintervention (*n* = 100).

**Table 1:** Distribution of studied nurses related to their characteristics (*n* = 100).

Items	*N*	%
Age:		
20–<25	68	68
25–30	17	17
>30	15	15
Mean (SD)		
	25.26 (4.78)	
Experience:		
<1 year	54	54
1-5 years	38	38
>5 years	8	8
Qualification:		
Diploma	6	6
Bachelor	84	84
Postgraduate	10	10
Nationality:		
Saudi	92	92
Non-Saudi	8	8
Training courses about innovation:		
Yes	38	38
No	62	62

**Table 2:** Distribution of studied nurses related to their knowledge about innovation pre- and postintervention (*n* = 100).

Domains	Pre		Post		Chi-square	*p* value
	Correct	Incorrect	Correct	Incorrect		
Concept of innovation standard “4 items”	22	78	69	31	9.868	<0.01^∗∗^
Benefits of innovation standard at nursing “3 items”	19	81	83	17	11.231	<0.01^∗∗^
Factors affecting innovation standard at nursing “3 items”	23	77	78	22	12.571	<0.01^∗∗^
Principle achievement of innovation standard strategy “3 items”	20	80	86	14	14.671	<0.01^∗∗^
Ways of achievement of innovation standards “4 items”	17	83	72	28	13.901	<0.01^∗∗^

**Table 3:** Distribution of studied nurses related to their individual innovative scale pre- and postintervention (*n* = 100).

Domains	Pre		Post		*t*-test	*p* value
	Mean	SD	Mean	SD		
Opinion leadership	8.96	2.01	14.32	3.16	6.987	<0.01^∗∗^
Openness to experience	5.03	1.78	10.08	2.31	7.664	<0.01^∗∗^
Resistance to change	9.08	2.60	13.99	2.87	6.302	<0.01^∗∗^
Cautiousness	2.33	0.98	4.50	1.01	7.099	<0.01^∗∗^
Risk-taking	2.51	0.86	4.87	0.76	8.312	<0.01^∗∗^

**Table 4:** Correlation between studied variables preintervention.

		Total knowledge	Individual innovative scale	Total attitude
Total knowledge	*r* *p*		0.601 <0.01^∗∗^	0.564 <0.01^∗∗^
Individual innovative scale	*r* *p*			0.537 <0.01^∗∗^
Total attitude	*r* *p*			

**Table 5:** Correlation between studied variables postintervention.

		Total knowledge	Individual innovative scale	Total attitude
Total knowledge	*r* *p*		0.577 <0.01^∗∗^	0.498 <0.01^∗∗^
Individual innovative scale	*r* *p*			0.601 <0.01^∗∗^
Total attitude	*r* *p*			

## Data Availability

The data used to support the findings of this study are included within the article.

## Additional Points

*Recommendation*. (1) On-the-job training program for nurses about innovative skills. (2) Further study to assess the barriers of applying innovative skills. (3) Further education with all healthcare workers who are involved in the care of patients in order to reinforce innovative behavior.
